# Risk Analysis of Textile Industry Foreign Investment Based on Deep Learning

**DOI:** 10.1155/2022/3769670

**Published:** 2022-01-10

**Authors:** Jingyi Liu, Jiaolong Li

**Affiliations:** ^1^School of Art and Design, South-Central University for Nationalities, Wuhan 430074, China; ^2^Department of Mathematics and Quantitative Economics, School of Statistics and Mathematics, Zhongnan University of Economics and Law, Wuhan 430073, China

## Abstract

With the decline of China's economic growth rate and the uproar of antiglobalization, the textile industry, one of the business cards of China's globalization, is facing a huge impact. When the economic model is undergoing transformation, it is more important to prevent enterprises from falling into financial distress. So, the financial risk early warning is one of the important means to prevent enterprises from falling into financial distress. Aiming at the risk analysis of the textile industry's foreign investment, this paper proposes an analysis method based on deep learning. This method combines residual network (ResNet) and long short-term memory (LSTM) risk prediction model. This method first establishes a risk indicator system for the textile industry and then uses ResNet to complete deep feature extraction, which are further used for LSTM training and testing. The performance of the proposed method is tested based on part of the measured data, and the results show the effectiveness of the proposed method.

## 1. Introduction

With the slowdown of China's economic growth rate and changes in the growth model, the original crude corporate model has become unsustainable [1–4]. It has become a matter of course for the people to increase their consumption expectations based on the continuous improvement of living material standards. As a dual-intensive industry of labor and capital, the development of the textile industry plays a key role in the development of China's economy and guarantees the level of employment. Compared with other industries, the textile industry has the characteristics of long process, wide distribution, large number of employees, intensive capital, obvious geographical concentration, and high export ratio. These characteristics have brought the complexity and high risk of China's textile industry. Since the Sino-US trade friction in 2018, the textile industry as the business card of China's manufacturing industry has been frequently hit. The list of additional tariffs imposed by the United States includes textile-related products, which has had a considerable impact on the Chinese textile industry. As an important part of China's foreign investment, scientifically conducting investment risk analysis in the textile industry plays an important role in improving economic benefits.

After years of development in the study of economic forecasting methods, a large number of forecasting models have emerged [5–15]. These models are divided into two categories: one is based on time series mainly including moving average and trend extrapolation and the other is based on causality, mainly including regression analysis, Markov prediction, and artificial neural network. In addition, the development of deep learning makes the fitting of complex systems more accurate. There are many studies on macroeconomic forecasts at home and abroad. Traditional economic forecasting methods, such as ARIMA and linear regression, have great limitations. ARIMA requires time series data to be stable. The linear regression is poor in fitting complex nonlinear systems. Aiming at the complex nonlinear relationship in macroeconomic forecasting, the neural network model with strong ability to fit nonlinear systems has become a hot spot in the research of macroeconomic forecasting all over the world. There are many studies on the use of BPNN to establish prediction models. Literature [6] built a transmission line project cost prediction model based on BPNN, which could accurately estimate the project cost using a small number of samples. Therefore, it was suitable for comparing the pros and cons of the project in the early stage. Literature [9] combined with the Radial Basis Function (RBF) neural network and unbiased gray model (GM) established a gray RBF neural network prediction model. Through the predictive analysis of fiscal revenue data, it is found that training with this model not only has a fast convergence rate but also strong ability and high model accuracy. Literature [13] proposed a hybrid radial basis neural network, which integrated ridge regression, regression numbers, and radial basis neural networks. It was proved by experiments to predict the daily average trend of stock indexes. This network had a good effect when there are complex nonlinear relations between variables and mutual dependence. After years of research and development, artificial neural networks and their various improved models still cannot completely get rid of the defect that they tend to fall into local minimums and cannot reflect the timing relationship between samples [16–24]. However, this timing relationship is common in the economic field, and predictive analysis is of great help. At the same time, long short-term memory (LSTM) in deep learning shows an excellent ability to process time series data in the field of prediction. Literature [18] combined the trend data of steel transaction prices in recent years and trained the LSTM model. This work was compared and analyzed with the support vector regression model and found that the LSTM neural network can more accurately predict the price trend of steel. Literature [20] used deep learning for several years of the Gross Domestic Product (GDP) data in China to establish a prediction model, and the results show that the prediction accuracy based on deep learning was significantly higher than that of ARMA, LR, and exponential regression. Literature [23] aimed at the random and nonlinear characteristics of traffic flow using LSTM and Gated Recurrent Unit (GRU) neural network methods to predict short-term traffic flow. The experiments had proved that the deep learning methods based on recurrent neural network LSTM and GRU performed much better than the ARIMA models and some other methods [25–29].

Based on the existing methods, this paper proposes a textile industry foreign investment risk prediction method by combination of LSTM and ResNet [30–33]. First, an indicator system is established for investment risks in the textile industry, and feature vectors are constructed to describe the risk levels in the current state. On this basis, ResNet is used to perform further feature learning on the constructed index feature quantity to obtain deep features with stronger descriptive ability. As a reliable deep learning prediction method, LSTM predicts the characteristics learned by ResNet and obtains the current risk representation. So, the current risk status of foreign investment in the textile industry can be judged. In the experiments, the proposed method is tested and verified with part of the data obtained publicly, and the results showed the effectiveness of the proposed method.

## 2. Basic Theory

### 2.1. LSTM

LSTM network is a model of memory cell network structure proposed by Hochreiter to solve the gradient explosion and gradient disappearance phenomenon that occurs when the recurrent neural network is processing relatively long time series data. It is introduced into the cell on the basis of Recurrent Neural Network (RNN). The threshold structure for judging whether the information meets the requirements is used to control the accumulation speed of information—input gate, forget gate, and output gate—so as to use this structure to memorize and update new information and solve the problem of long-term dependence. As shown in Figure 1, each LSTM neuron is composed of cell states, namely, long-term state *c*_*t*_ and short-term state *h*_*t*_, input gate *i*, forget gate *f*_*t*_, and output gate *o*_*t*_.

The so-called cell state is a container for storing information. Through the process control of input gate, forget gate, and output gate, the information in the container is gradually increased, decreased, changed, and output. In each neural unit, the cell state undergoes the forgetting process of the forget gate, the input process of the input gate, and the process of outputting information to the output gate. The input gate is to copy and process the input information of the current neural unit. It consists of two parts: the sigmoid function independently chooses which information to update and the tanh function adds the constructed brand new vector to the current cell state to construct a new state. The realization formula is as follows:

(1) $$\begin{array}{c} \left\{\begin{array}{c} i_{t}=\sigma \left(w_{xi}x_{t}+w_{hi}h_{t-1}+b_{i}\right),\\ {\tilde{c}}_{t}=\phi \left(w_{xc}x_{t}+w_{hc}h_{t-1}+b_{c}\right). \end{array}\right. \end{array}$$

The main function of the forget gate is to determine which information needs to be discarded in the current state. *f*_*t*_=1 means that the information is completely retained; *f*_*t*_=0 means that the information is completely discarded. The realization formula of *f*_*t*_ is as follows:

(2) $$\begin{array}{c} f_{t}=\sigma \left(w_{xf}x_{t}+w_{hf}h_{t-1}+b_{f}\right). \end{array}$$

The output gate mainly controls the output information of the current hidden state. The realization formula is as follows:

(3) $$\begin{array}{c} \left\{\begin{array}{c} h_{t}=o_{t}\tanh\left(c_{t}\right),\\ c_{t}=i_{t}{\tilde{c}}_{t}+f_{t}c_{t-1},\\ o_{t}=\sigma \left(w_{xo}x_{t}+w_{ho}h_{t-1}+b_{o}\right). \end{array}\right. \end{array}$$

In equation (3), *h*_*t*−1_ is the output at the time *t* − 1; *w*_*xi*_, *w*_*xc*_, and *w*_*xo*_ are the matrix weight parameters for the input vector *x*_*t*_ the at the time *t*, respectively; *w*_*hi*_, *w*_*hc*_, and *w*_*ho*_ represent the weight matrix parameters of the hidden layer vector *h*_*t*−1_ at the time *t* − 1; and *b*_*i*_, *b*_*c*_, *b*_*f*_, and *b*_*o*_ represent the bias vector parameters.

Finally, the back propagation through time (BPTT) algorithm can be used to optimize the parameters of the LSTM model to obtain a reliable prediction model.

### 2.2. ResNet

As the number of deep neural network layers continues to increase, the learning ability of the network becomes stronger and stronger. However, the convergence speed of the relative network will slow down, and the gradient will disappear during the propagation process, making it impossible to effectively adjust the weights of the previous network layers. In the traditional convolutional neural networks (CNNs), except for the first layer, the input of each layer is derived from the output of the previous layer. The ResNet adopts a skip structure so that the deep residual network can directly cross the middle layers. The parameters are passed to the subsequent layers, which reduces the complexity of the network, solves the degradation problem of the deep-level network, and promotes the improvement of network performance.

The network structure of the residual neural network is shown in Figure 2. The network draws on the idea of cross-layer connection of high-speed networks. In the residual unit structure shown in Figure 2, *x* is the input of the network; *H*(*x*) is the optimal solution mapping; and *F*(*x*) represents the residual term and directly passes the input *x* to the output as the initial result to get the output *H*(*x*)=*F*(*x*)+*x*. When *F*(*x*)=0, *H*(*x*)=*x* is an equal mapping. The training goal of ResNet is to make the residual term *F*(*x*)=*H*(*x*) − *x* close to zero. It is easier to let *F*(*x*)=0 than *H*(*x*)=*x*. The updated parameters using *F*(*x*)=0 can converge faster. Compared with the network model that does not adopt the skip structure, the residual network of this structure has clearer input data and can retain the accuracy of the data to the greatest extent.

## 3. Risk Assessment Method

### 3.1. Index System

The purpose of financial early warning indicators is to detect the possible financial risks of the enterprise in advance and to rate the risks. Therefore, when selecting indicators, you should choose indicators with the nature of capability evaluation and risk evaluation. Therefore, based on relevant domestic and foreign research results, this article selects the total return on net assets, net sales interest rate, net operating cash flow/debt, and operating activities from five aspects: profitability, operating ability, development ability, debt solvency, and cash flow ability. A total of 10 financial indicators including net cash flow growth rate, net asset growth rate, total asset growth rate, accounts receivable turnover rate, current asset turnover rate, asset-liability ratio, and asset-liability ratio are statistically analyzed. Based on the data indicators of the textile industry's foreign investment, the feature vectors of these 10 indicators can be constructed accordingly, which can be used for subsequent risk prediction and evaluation.

### 3.2. Evaluation Process

This paper builds a ResNet-LSTM-based textile industry foreign investment risk analysis model based on the previous discussion. The proposed method makes full use of the advantages of ResNet and better retains the attributes of the original data so as to effectively solve the problem of extracting the characteristics of financial risk data in the textile industry. Using the advantages of LSTM in data prediction, the accuracy of risk prediction is improved through ResNet's deep features. The basic flow chart of the method in this paper is shown in Figure 3, and the specific steps are described as follows:

1. Based on the historical data set of the textile industry's foreign investment, the feature vector is constructed according to the established index system.
2. ResNet is used for deep feature extraction to further optimize the feature vector.
3. In the training phase, the deep features extracted by the optimized ResNet are input into the LSTM network, and the unique characteristics of the memory unit structure of the LSTM network are used to establish a prediction model.
4. In the testing phase, the investment financial data set of the current data is input to the established LSTM prediction model, and the current risk assessment result is output.

### 3.3. Evaluation Index

Assuming the predicted value as $\hat{y}=\left\{{\hat{y}}_{1},{\hat{y}}_{2},\ldots ,{\hat{y}}_{n}\right\}$ and the true value as *y*={*y*_1_, *y*_2_, ⋯, *y*_*n*_}, the root mean square error (RMSE), mean absolute percentage error (MAPE), and mean accuracy (MA) are used as the evaluation indicators of the perdition model. The definitions of the three indexes are as follows:

(4) $$\begin{array}{c} \text{RMSE}=\sqrt{\frac{1}{n}\overset{n}{\underset{i=1}{\sum }}{\left({\hat{y}}_{i}-y_{i}\right)}^{2}},\\ \text{MAPE}=\frac{1}{n}\sum_{i=1}^{n}\left|\frac{\left({\hat{y}}_{i}-y_{i}\right)}{y_{i}}\right|\times 100\%,\\ \text{MA}=1-\text{MAPE.} \end{array}$$

In the formula, the smaller the RMSE value, the closer the predicted value to the true value, the higher the accuracy of the prediction. MAPE and MA evaluate the predictive power of the model. The smaller the MAPE and the larger the MA, the better the prediction effect of the model.

## 4. Experiment and Analysis

### 4.1. Data Set and Comparison Method

In order to test the performance of the proposed method, this paper obtained 380 historical financial data of China's textile industry foreign investment through public channels. According to the financial risk measurement index system in the previous works, the corresponding feature vectors are constructed, respectively. Then, the method of combining ResNet and LSTM is used for risk prediction analysis, and RMSE and MA indicators are used to evaluate the performance of the method. While testing the method in this paper, some existing methods are selected for comparative analysis, including the method based on support vector machine (SVM), the method based on BP network, and the method based on LSTM.

## 5. Results and Analysis

The selected investment data are tested using the proposed method, and the performance of the method in this paper and the comparison methods is as shown in Table 1. According to the results, the performance of the method in this paper is the best among the four types of methods, reflecting its performance advantages. Among the three types of comparison methods, LSTM has the best performance, indicating its significant advantages in data prediction. BP network also has certain advantages over SVM, which shows the advantages of neural network. In particular, comparing the proposed method with LSTM shows that this paper further introduces ResNet for deep feature learning, which further improves the final prediction performance.

Therefore, by using the comprehensive evaluation of RMSE and MAPE two indicators, the proposed method has advantages in predicting the risk of foreign investment in the textile industry.

In the actual process, due to the influence of market bands and other political and economic factors, certain errors may occur in the prediction model. To this end, this paper applies a certain degree of noise to the experimental data to reflect the volatility of economic data. On this basis, MA was used as the basic evaluation index to test the performance trend of various methods, and the results are shown in Figure 4. It can be seen from the figure that the performance of various methods is degraded to a certain extent due to the influence of noise. In comparison, the method in this paper can maintain the best prediction performance under different noise interference conditions, thereby further improving its performance advantages.

## 6. Conclusion

Scientific analysis of the risk of foreign investment in the textile industry is conducive to identifying the investment direction and investment market and obtaining the greatest rate of return. Aiming at the problem of predicting the risk of foreign investment in the textile industry, this paper comprehensively uses two deep learning models, ResNet and LSTM. ResNet is used for deep feature learning to further optimize the index system of risk prediction. As an accurate and efficient prediction model, LSTM predicts the deep features learned by ResNet and obtains risk prediction results. Part of the measured data is used to verify and analyze the proposed method, and the result proves the performance advantage of the proposed method. Compared with the method directly using LSTM, the proposed can bring performance improvement owing to the merits of ResNet. In the future, more suitable deep learning models can be further developed to improve the accuracy of the prediction model.

## Figures and Tables

**Figure 1:** Basic structure of LSTM.

**Figure 2:** Illustration of residual network unit.

**Figure 3:** Prediction of investment risk based on LSTM and ResNet.

**Figure 4:** Performance of different methods under noises.

**Table 1:** Comparison of prediction performance of different methods.

	RMSE	MA (%)
Proposed	0.14	97.3
SVM	0.21	95.6
BP	0.18	96.1
LSTM	0.15	96.8

## Data Availability

The dataset can be accessed upon request.
